# Antigallbladder Carcinoma Activity Analysis of a New Nanometer Drug Delivery System Based on Data Acquisition

**DOI:** 10.1155/2022/9538051

**Published:** 2022-07-06

**Authors:** Weidong Li, Zhiye Liu, Yuanyuan Liu, Lei Qian, Zhiyong Zhang, Lei Nie, Xiusheng Qu

**Affiliations:** ^1^The First Affiliated Hospital of Jiamusi University, Department of Emergency, Jiamusi 154000, China; ^2^The First Affiliated Hospital of Jiamusi University, Department of Radiotherapy and Chemotherapy, Jiamusi 154002, China; ^3^The School Hospital of Jiamusi University, Jiamusi 154000, China; ^4^The First Affiliated Hospital of Jiamusi University, Department of Post Graduation Continuing Education, Jiamusi 154000, China; ^5^The First Affiliated Hospital of Jiamusi University, Department of Pediatrics, Jiamusi 154000, China

## Abstract

In order to solve the problem of the application of data acquisition in the new nanometer drug delivery system of microscope, a research of antigallbladder carcinoma activity analysis was proposed. Gallbladder carcinoma (GBC) is a common malignant tumor in biliary tract diseases. Due to the lack of specific clinical manifestations in the early stage, GBC has the shortcomings of the hidden onset, the difficult diagnosis, and the high misdiagnosis rate. GBC ranks in the top position among the most common tumors of the digestive system worldwide. The preoperative diagnosis rate is low, and the incidence of accidental gallbladder carcinoma is gradually increasing. Domestic gallbladder carcinoma related to cholecystectomy is not sensitive to radiotherapy and chemotherapy. Surgical resection is still the only effective method for the treatment of accidental gallbladder carcinoma.

## 1. Introduction

With the development of nanotechnology, many problems have been solved successfully in carcinoma treatment. Multidrug resistance is a major problem in carcinoma treatment. The third generation of nanodrugs with multiple functions has strong ability in drug delivery, protection, and specific transport, which can overcome the problem of drug resistance to a large extent. Moreover, it can improve the efficacy of combination therapy and achieve controlled release of drugs, thus further overcoming drug resistance. Carcinoma diagnosis is another challenge. Traditional carcinoma diagnosis is based on a single indicator and is often influenced by the patient's physical condition, drug response, and immune status. It is helpful for carcinoma diagnosis to identify a small number of tumor-specific molecular, genetic, or transcriptome markers in blood and tumor tissue. Currently, several nanoparticles have been developed for both diagnosis and treatment of carcinoma. Tumor metastasis is an important cause of death in carcinoma patients. At present, there is no effective treatment strategy for tumor metastasis and there are no appropriate means to detect the status of tumor metastasis. The complex physical environment of the patient is a major obstacle to the development of effective treatment. Nanotechnology can specifically target tumors in different organs, which offers an opportunity to treat metastases. With the development of sequencing technology, genes in tumor tissues have individual differences and mutations. Individual therapy has become the main direction of carcinoma treatment in the future. The development of multifunctional nanoparticles provides an important guarantee for the personalized treatment of carcinoma.

## 2. Literature Review

The new nanometer drug delivery system mainly includes magnetic nanoparticles, ultrasonic mediated nanodrug delivery system, and bionic drug delivery system. At the same time, the new nanoparticle drug delivery system has also been applied in the diagnosis and treatment of epilepsy. Gallbladder carcinoma is the most common malignant tumor of the gallbladder, the incidence of which is increasing year by year. It usually occurs in people over 50 years old. At present, the prognosis of gallbladder carcinoma is still very poor and many patients die within 1 year [1].

The research conducted by Mehrotra et al. showed that, combined with laser irradiation, the way that the vein was injected with HpD could treat various tumors [2]. So far, some preclinical and clinical researches around the world showed that PDT was a minimally invasive treatment for carcinoma, which was effective. The role of the Bcl-2 gene in tumor apoptosis is still controversial. Lin et al. pointed out that overexpression of Bcl-2 could inhibit apoptosis induced by various stimuli [3]. Gautam et al. reported that TPC4-PDT inhibited apoptosis of Chinese mouse ovarian carcinoma cells overexpressing Bcl-2 [4]. Geng et al. proposed that multiple photosensitively-mediated photodynamic effects could downregulate the expression of Bcl-2 protein in mouse leukemia cell line L1210, but had no effect on Bax protein expression [5]. Abeer et al. proposed the main advantages of PDT in the treatment of gallbladder carcinoma. The biggest advantage lay in its high selectivity to tumor cells, including two selection processes. One was that photosensitivities were selectively enriched in tumor cells, and the other was that light sources were selectively irradiated to the tumor area [6]. Among the photosensitizers Liu, Y. B. used in the photodynamic therapy of gallbladder cancer, Photosan and photoporphyrin as photosensitizers of hematoporphyrin derivatives, which are most widely used at present [7]. Kim et al. proposed that nanotechnology was used to improve the photochemical efficiency of photosensitizer, improve its water solubility and bioavailability, increase the concentration of effective photosensitive drugs in tumor tissues, improve the photodynamic therapy effect of gallbladder carcinoma, and reduce the toxic and side effects of photosensitive drugs [8].

On the basis of some current researches, the research on antigallbladder carcinoma activity analysis was proposed. The nanometer technology principle was that, in the nanosize range, new materials with specific functions were made by manipulating individual atoms and molecules directly. The physical and chemical properties of substances changed as they rearranged atoms down to the nanometer scale. Small size effect, surface effect, quantum size effect, and macroscopic tunnel effect appeared. The new features of the nanoparticles appeared, which were different from the conventional material, such as good photochemical and photoelectromagnetic properties; solubling in water easily; and high bioavailability. Nanoparticles had small size and large surface area. The number of surface atoms, surface energy, and surface tension increased sharply with the decrease of particle diameter. The surface atoms lacked neighboring atoms and had many dangling bonds, which were unsaturated and easy to modify biomolecules on their surface. Nanotechnology was utilized to improve the photochemical efficiency of photosensitizer and its water solubility and bioavailability. The concentration of effective photosensitive drugs in tumor tissues could be increased. The photodynamic therapy effect of gallbladder carcinoma could be improved and the toxic and side effects of photosensitive drugs could be reduced [9].

## 3. Analysis of the Antigallbladder Carcinoma Activity of the New Nanometer Drug Delivery System Based on Data Collection

### 3.1. New Nanometer Drug Delivery System

Magnetic nanoparticles (MNP) are a kind of special particles composed of magnetic iron oxide nanoparticles and other metal nanoparticles. Drug-carrying magnetic nanoparticles usually contain drugs, magnetic nanoparticles, and skeleton materials. A core-shell structure is usually adopted. Magnetic nucleus is for targeting. MNP has the shell with affinity and biocompatibility, which is the drug wrapped in the particle or bound to the shell layer of molecules. Magnetic targeting of drug-carrying nanoparticles enters the human body by means of injection or mouth.

A certain intensity magnetic field is exerted on the outside of the lesion site. By the inductive effect of magnetic field, the phagocytosis of macrophages can be avoided in the reticuloendothelial system. The magnetic drug-carrying nanoparticles can be aggregated to the lesion site, and then the drug can be localized and released in a controlled manner. Magnetic targeted drug delivery can significantly reduce drug dose and realize the unification of high efficiency and low degree of drug delivery system. Magnetic nanoparticles have both nanometer effect and superparamagnetism, which can be used as gene delivery vector materials after polymer modification. Chitosan has basic amino functional groups that can aggregate nucleic acids to form stable complexes that protect DNA from nuclease degradation. As a biodegradable natural polymer material, chitosan has very weak toxicity. Composite magnetic nanoparticles formed by chitosan-coated magnetic nuclei are an excellent nonviral gene carrier material [10].

MNP is used in targeted drug delivery, known as magnetic drug targeting. Magnetic targeted carrier (MTC) is a combination of MNP and the drug to be delivered by covalent or noncovalent means. Since the particles themselves are magnetic, the targeting ability of MTC can be improved by applying external magnetic field to the lesion site. Since the secondary magnetic components (such as Fe3O4) contained in MTC are relatively fixed with drug components, the amount of drug entering the target site can also be traced by MRI. Similar to conventional nanoparticles, MTC can also be remodified on its surface with small peptide groups with targeted function, resulting in the formation of multifunctional MTC. Monocytes and neutrophils express integrin receptors that selectively bind to arginine-glycine-aspartate tripeptides (RGD). Researches showed that GD-modified magnetic liposomes (liposome-coated Fe3O4) can be selectively ingested by monocytes/neutrophils in blood circulation to avoid phagocytosis by macrophages in the liver and other tissues. Magnetic fields are added to external inflammatory areas or lesion sites. Since liposomes ingested by cells are magnetic, it can make the absorbed magnetic liposome cells gather to the target site under the action of the magnetic field, which can be used for brain-targeted drug delivery [11].

### 3.2. The Development Stage of Nanoscale Anticarcinoma Weapons

The first generation nanomedicine can accumulate at the tumor site through the hyperpermeability of the tumor site blood tube, but it does not specifically target the tumor. These nanocarriers can prolong the half-life of drugs and reduce the toxic side effects of drugs. The first-generation drugs have been approved by the US Food and Drug Administration for the clinical carcinoma treatment. The second generation of nanomedicine can actively target tumor cells, which can better improve drug delivery and increase its aggregation at the tumor site. The drug can be taken up more by tumor cells, thus improving the therapeutic effect. At the same time, some proteins with high expression on the surface of tumor cells can be used as targets to design targeted nanodrugs. Many nanodrugs with specific targeting ligands are already in clinical trials and their success holds promise for carcinoma treatment. The third generation of nanomedicines has multiple skills that can be used for early detection, diagnosis, prevention, and treatment of tumors. It has the ability of precise pharmacokinetic control, which can improve the half-life of the drug and achieve controlled release of the drug, thus enhancing its efficacy and greatly reducing the toxic side effects. At the same time, the combination of multiple drugs can be realized, so that the drugs can be released in the tumor site and carry out a joint attack on carcinoma. The third generation of nanoparticles has great advantages in drug delivery, tumor imaging, and gene therapy [12].

### 3.3. Application of New Nanometer Drug Delivery System in Gallbladder Carcinoma

At present, the diagnosis of gallbladder carcinoma is mainly based on clinical symptoms, electroencephalogram, and imaging examination. The cause diagnosis of gallbladder carcinoma mainly depends on the genes check, but the specific gene is not found for many gallbladder carcinomas. Especially refractory gallbladder may be related to gene mutation and targets (ion channels and receptors) desensitization and local drug transporter high expression, which also makes the etiological diagnosis of gallbladder carcinoma more difficult [13].

Magnetic nanoparticles in new nanodrug delivery systems have great potential in the diagnosis and targeted therapy of brain diseases. It is found that magnetic nanoparticles can be used as a new NMR contrast agent for disease diagnosis. Researches have shown that long-circulating superparamagnetic Fe3O4 can better delineate the boundaries of brain tumors and surrounding normal tissues than traditional chelating contrast agents. The ultrasonic mediated nanodelivery system improves the accuracy of MRI targeting specific areas by injecting standard microbubble contrast agents intravenously and enriching BBB in the parenchymal region through a series of mechanical, chemical, and thermal effects.

Currently, AEDs in use can be got by BBBS, but most of them are substrates for external pump proteins such as P-gp on BBBS. Therefore, they can be pumped back into the bloodstream from the brain, resulting in poor or resistant treatment of gallbladder carcinoma with conventional AEDs. The new nanodrug delivery system can enhance the concentration of drugs reaching targeted lesions through magnetic and aggregation ultrasound methods, while the bionic drug delivery system can reduce the phagocytosis of macrophages due to the same cellular mechanism in vivo, which plays a better role in drug delivery [14].

### 3.4. Clinical Manifestations of Gallbladder Carcinoma

Early gallbladder carcinoma is often without obvious clinical symptoms. The so-called early gallbladder carcinoma is found mostly in other operations by accident. Part of early gallbladder carcinoma is combined with gallstone, which is found when cholecystolithiasis resection is conducted. The main clinical manifestations of most gallbladder carcinomas are epigastric pain, nausea, vomiting, jaundice, and right epigastric mass due to large tumor compression on the bile duct. There is no specific tumor marker for gallbladder carcinoma and CA19-9 can only be used as a reference indicator [15].

### 3.5. Treatment Results of Gallbladder Carcinoma

Once the diagnosis of gallbladder carcinoma is made, surgical resection is preferred. For the range of surgical resection, radical resection of stage I and II gallbladder carcinoma includes simple gallbladder resection, expanded gallbladder carcinoma resection, and regional lymph node dissection. Enlarged resection of gallbladder carcinoma in stage III and IV is feasible, including partial hepatic lobectomy and sometimes pancreaticoduodenectomy. By analyzing the data of patients undergoing surgery in this group, it was found that cholecystectomy or radical cholecystectomy was feasible for stage I and II gallbladder carcinoma, including skeletonization of the biliary trigone, hepatoduodenal ligament, and wedge resection of the liver with a depth of 2 cm in the gallbladder bed, which was with a good prognosis. Expanded resection of gallbladder carcinoma had a poor prognosis even if the resection scope was wide (including extrahepatic bile duct, colon, duodenum, and liver IVV) [16]. A small number of patients survived for a long time when the right lobe of the liver was enlarged for gallbladder carcinoma. The long-term survival of the patients was mainly due to completing tumor resection without lymph node metastasis, which was combined with radiotherapy. The efficacy of portal vein resection or pancreaticoduodenectomy was not good, and there was no substantial improvement in the condition of unresected patients. Radiotherapy and interventional therapy could only be used as adjuvant therapy, and the clinical efficacy of radiotherapy or interventional therapy was not obvious. In conclusion, radical surgery was effective for gallbladder carcinoma at stages I and II, while radical resection was feasible for gallbladder carcinoma at stages III and IV. Radical surgery is difficult for patients with liver metastasis, peritoneal metastasis, or para-aortic lymph node metastasis, and radiotherapy and interventional therapy could only be used as adjuvant therapy. At the same time, the level of early diagnosis of gallbladder carcinoma should be improved to increase the long-term survival rate of patients with gallbladder carcinoma [17].

As for cholecystectomy, laparoscopic surgery is the first choice. If the patient is combined with absolute or relative contraindications of laparoscopic surgery, open surgical resection is chosen. If there are surgical accidents or difficult operations in laparoscopic surgery, open surgery is needed halfway. The gallbladder triangle is dissected carefully. The gallbladder artery and cervical duct are ligated and dissociated. The complete cholecystectomy is performed anterograde or retrograde. During the operation, the integrity of the gallbladder should be ensured to prevent bile or stone overflow. For patients with suspected intraoperative gallbladder carcinoma, the rapid intraoperative frozen section was performed.

As for radical operation for gallbladder carcinoma, the liver tissues of the gallbladder and gallbladder bed which are lymph nodes, nerves, and connective tissue in the hepatoduodenal ligament are removed. The portal vein, hepatic artery, and common bile duct should be bare. The parahepatic artery lymph nodes, celitoneal trunk lymph nodes, retroportal vein, and retropancreatic duodenal lymph nodes are removed.

As for expanded radical resection of gallbladder carcinoma, the specific surgical method depends on the local infiltration and metastasis of the tumor. Extrahepatic bile duct reconstruction, enlarged right hepatectomy, pancreaticoduodenectomy, and right colectomy are generally added on the basis of radical resection of gallbladder carcinoma [18].

## 4. Discussion

Once gallbladder carcinoma is diagnosed, radical surgical resection is still the preferred method. However, due to the lack of specific clinical symptoms in the early stage, GBC is mostly diagnosed in the middle and late stage. The chance of radical treatment is lost, resulting in a poor prognosis [19]. There is no clear etiology of gallbladder carcinoma, but epidemiology shows that it is related to the presence of gallstones [20].

Based on the gallstones in the research, the occurrence of gallbladder carcinoma still accounts for a large proportion, which may be related to the long-term physical stimulation of gallstones and chronic inflammatory stimulation of mucosa, especially the irregular thickening of the gallbladder wall. So, the occurrence of gallbladder carcinoma should be warned [21]. For the treatment of gallbladder carcinoma, surgical resection should be used as the main comprehensive treatment measures. At present, simple resection is enough for patients at Tis and pT1a stages, which has been recognized by the majority of scholars. The current treatment for pT1b patients is controversial. Some scholars believe that cholecystectomy alone is the purpose of treatment. Some people believe that radical gallbladder carcinoma can improve the 5-year survival rate of patients. For patients at this stage, radical surgery is still preferred, which is consistent with the results of the research. The theoretical basis of radical operation for pT1b stage is the characteristic of lymph node metastasis of gallbladder carcinoma. Lymph node metastasis can occur early when the invasion gets to gallbladder wall muscle layer. Due to the large number of complications and high surgical risks, whether patients at pT2 and pT3 stages should undergo extended radical surgery can be considered individually and comprehensively according to the size of lesions, infiltration, metastasis, and surgical skills of doctors and the patient's conditions [22].

In order to reduce the occurrence of accidental gallbladder carcinoma, clinical attention should be paid to the high-risk groups of gallbladder carcinoma. The high-risk groups of gallbladder carcinoma include older women, the patients whose preoperative imaging findings were gallbladder-filled calculi or Mirizzi syndrome, the patients whose nature and regularity of abdominal pain changed obviously, the patients whose gallbladder adenomyosis or single polyp is larger than 1 cm, and patients who suffer from gallbladder atrophy, porcelain, or thickening. Intraoperative routine cholecystectomy and rapid freezing examination are performed. Postoperative attention should be paid to paraffin pathological results to reduce the occurrence of UGC. With the continuous development of perioperative management, surgical techniques, and surgical instruments in recent years, the number of cases of radical surgical resection for gallbladder carcinoma at the middle or late stage has increased and the complications have decreased [23].

In a word, gallbladder carcinoma has a high degree of malignancy, rapid progression, and poor prognosis. Early diagnosis and early operation are the keys to improve the survival of gallbladder carcinoma [24]. Ultrasound, CT, and other imaging examinations are the main methods of preoperative diagnosis of gallbladder carcinoma. Appropriate surgical methods should be selected according to the tumor stage to prolong the lifetime and improve the prognosis [25].

### 4.1. Analysis Process of Biological Information Data

In the information analysis process, the preliminary data filtering is completed by removing the connectors at both ends of reads, removing low-quality reads, and removing contamination. Clean reads are obtained, and the sequence length distribution and the common sequences among samples are counted. Clean reads are classified and annotated to obtain the composition and expression information of various microRNAs in the samples. After all microRNA fragments are annotated, the remaining annotated fragments are used to predict new miRNA. The process of biological information data analysis is shown in Figures 1 and 2.

## 5. Conclusion

The development of nanotechnology has changed people's lives, which will benefit people in diagnosing and treating diseases in the future. Nanometer drug delivery system is a promising research direction for carcinoma treatment, which will provide a new therapeutic approach for carcinoma treatment. With the development of nanotechnology research, nano anticarcinoma weapons will push carcinoma treatment into a new era. However, the development of nanocarcinoma weapons depends not only on the innovation of nanotechnology but also requires a sufficient understanding of the molecular biological mechanism of carcinoma. Only in this way can we find the true weakness of carcinoma and design more effective drugs to win the modern war on carcinoma. Of course, before drugs are used in clinical patients, a large number of clinical researches are needed to investigate the safety and effectiveness of drugs, so as to better solve the pain of carcinoma patients and bring hope to patients' families. The malignant degree of gallbladder carcinoma is high. The resection rate is low, and the overall prognosis is poor. Because the research on the pathogenesis of gallbladder carcinoma is not enough, surgical operation alone cannot achieve the goal of treatment. Therefore, the comprehensive treatment of gallbladder carcinoma should be paid attention to and emphasized, trying to improve the quality of life of patients and prolong their survival period. With further research on the mechanism of gallbladder carcinoma, photodynamic therapy is hoped to become an important means to break through the bottleneck of gallbladder carcinoma treatment in the future.

## Figures and Tables

**Figure 1:** Biological flow chart.

**Figure 2:** Analysis flow chart of biological information data.
